# Optical Coherence Tomography in Multiple Sclerosis and Neuromyelitis Optica: An Update

**DOI:** 10.1155/2011/472790

**Published:** 2011-06-02

**Authors:** Susana Noval, Inés Contreras, Silvia Muñoz, Celia Oreja-Guevara, Beatriz Manzano, Gema Rebolleda

**Affiliations:** ^1^HIV Unit, Ophthalmology Department, Hospital La Paz/Autónoma University School of Medicine, IdiPAZ, Madrid, Spain; ^2^Ophthalmology Department, Clinica Rementería, Hospital Ramón y Cajal, Alcalá de Henares University School of Medicine, Madrid, Spain; ^3^Ophthalmology Department, Hospital Universitari de Bellvitge, L'Hospitalet de Llobregat, Barcelona, Spain; ^4^HIV Unit, Neurology Department, Hospital La Paz/Autónoma University School of Medicine, IdiPAZ, Madrid, Spain; ^5^HIV Unit, Hospital La Paz/Autónoma University School of Medicine, IdiPAZ, Madrid, Spain

## Abstract

Optical coherence tomography (OCT) uses light interference patterns to produce a cross-sectional image of the retina. It is capable of measuring the unmyelinated axons of the retinal ganglionar cells as they converge on the optic disc. In a disease like multiple sclerosis (MS), in which axonal loss has been identified as an important cause of sustained disability, it may prove an invaluable tool. OCT has demonstrated that axonal loss occurs after each episode of optic neuritis and that the degree of axonal loss is correlated to visual outcomes. Furthermore, axonal loss occurs in MS even in the absence of inflammatory episodes, and the degree of this loss is correlated with the duration of the disease process, with more thinning as the disease advances and in progressive forms. Thus, OCT retinal nerve fiber layer measurements may represent an objective outcome measure with which to evaluate the effect of treatment.

## 1. Introduction

The optic nerve as it leaves the eye is the only tissue composed of unmyelinated axons which can be imaged directly. The retinal nerve fiber layer (RNFL) is made up of the axons of the retinal ganglionar cells that convey the visual information from the retina to the lateral geniculate nucleus; until they exit the eye, they do not acquire the protective myelin sheath. This extraordinary circumstance allows us to study the influence on isolated axons of several diseases. Ganglionar cells and their axons, besides being the main retinal component around the optic nerve (90% of retinal thickness) are also representative at the macula (30–35%). 

Both time-domain and spectral-domain optical coherence tomographies (OCT) use light interference patterns to produce a tomogram, or cross-section, through the layers of the retina. From this information, the OCT software constructs a two-dimensional (time-domain, TD-OCT) or three-dimensional (spectral-domain, SD-OCT) image of the retina and the optic nerve and is capable of measuring the different layers of the retina with a margin of error of 4–6 *μ*m. The reproducibility of RNFL and macular measures has been found to be excellent with SD-OCT in multiple sclerosis [1]. Multiple studies have provided information on the normal values for the RNFL thickness and have reported the RNFL loss that occurs after different pathologies that affect the optic nerve.

Axonal loss, in contrast to demyelination, is not reversible and is therefore an important cause of sustained disability. In patients diagnosed with multiple sclerosis, it has been demonstrated that axonal loss occurs in the early stages of the disease. This is one of the reasons that support the early use of neuroprotective drugs. Monitoring axonal loss has become a priority in multiple sclerosis and OCT as a sensitive, precise, and reproducible technique is acquiring increasing importance for both neurologists and ophthalmologists [2]. 

## 2. Isolated Acute Optic Neuritis

Optic neuritis is one of the manifestations of multiple sclerosis; it has been described as the second most frequent mode of presentation. The Optic Neuritis Treatment Trial (ONTT) has shown us that a patient diagnosed with a first episode of optic neuritis has a risk of 50% of developing multiple sclerosis in the following 15 years. The risk increases to 72% in those patients with at least one demyelinated lesion on magnetic resonance imaging (MRI) and decreases to 25% in those without lesions [3]. However, these data are not applicable to all patients, for example, in Asian populations MRI lesions are less frequently encountered [4]. 

### 2.1. Acute Changes in Anterior Optic Neuritis

Optical coherence tomography has a high sensitivity for detecting acute optic nerve oedema in anterior optic neuritis (Figure 1). Our study group performed one of the first prospective studies evaluating TD-OCT in acute optic neuritis. Twenty-three patients underwent a complete ophthalmological evaluation, including visual acuity (VA) measurement, automated static perimetry, and OCT at onset and periodically for six months. We found a statistically significant increase in initial mean RNFL thickness in anterior forms (166.30 *μ*m, SD 34.87 *μ*m) as compared to retrobulbar neuritis (98.60 *μ*m, SD 21.58 *μ*m), Doctoral thesis: “Study of optic neuritis with optical coherence tomography.” 

### 2.2. Axonal Loss

Following an initial episode of optic neuritis, OCT can detect axonal loss as a thinning of the RNFL, occurring mainly in the first three to six months (Figure 2). After this period, axonal loss stabilizes [5–7]. RNFL measurements obtained within the first eight weeks of optic neuritis may reflect the extent of optic disc and RFNL edema due to an acute bulbar or retrobulbar injury; whereas RNFL values obtained 3 or more months after ON may indicate the extent of axonal injury referable to the acute inflammatory event [7]. 

Prospective studies estimate that there is a 20 to 25% loss in the RNFL thickness when compared to the fellow unaffected eye (Table 1) [5, 6, 8]. The decrease is greater in Asian patients whose visual function is damaged more severely [4]. Most studies have been unable to demonstrate a significant thinning of the RNFL of the fellow eyes when compared to healthy controls [8–11]. 

Axonal loss affects diffusely the whole peripapillary RNFL, although the temporal quadrant is often the most affected. This loss may be detected as soon as two months after the event, when compared to the fellow eye and healthy controls [4, 7, 8]. Temporal thickness decreases between 25 and 34% [5, 8, 12]. This reflects a predominant affectation of the papillomacular bundle, which conveys the information from the fovea, the central macular structure mainly responsible for detailed visual and color functions. Therefore, macular volume is also mildly reduced in eyes that have suffered optic neuritis [13], especially in the nasal sectors of the macula [14]. Cutoff points of 51.5 *μ*m for the temporal RNFL thickness and 88.8 *μ*m for the average RNFL thickness have shown the highest sensitivity (0.72 and 0.60, resp.) and specificity (0.95 and 0.97, resp.) for differencing optic neuritis eyes from control eyes [8].

The optic nerve can become pale after an episode of optic neuritis. This pallor can be diffuse or located in the temporal quadrant and reflects the RNFL loss detectable with OCT. Because the temporal quadrant of the optic disc is relatively thinner than other quadrants, even diffuse atrophy may be perceived only as temporal pallor on exam. Our study group also found a mild increase in the cup to disc ratio of approximately 0.1 to 0.2 when compared to the fellow eye, in accordance with previous clinical observations [15, 16]. 

### 2.3. Visual Prognosis

Since RNFL loss after an episode of optic neuritis stabilizes after six months, most studies that analyze the relationship between axonal loss and visual outcome are performed at or after this time point. Costello et al. found that patients with incomplete visual recovery after optic neuritis suffer a greater RNFL loss and through regression analysis obtained a threshold of RNFL thickness (75 *μ*m) below which RNFL measurements predicted persistent visual dysfunction. This finding could be interpreted as a threshold effect whereby changes in RNFL thickness above 75 *μ*m are associated with minimal and clinically insignificant changes in visual field threshold sensitivity [5, 7]. In Costello's study, for RNFL values below 75 *μ*m, a 10 *μ*m decrease in RNFL thickness predicted a decrease of 6.83 dB in visual field mean deviation scores among affected eyes [7].

Visual fields represent a subjective method of measuring visual function, which requires active collaboration and attentiveness from the patient. Visual fields usually improve after a first episode of optic neuritis to normal or near normal levels. However, OCT often reveals subclinical permanent axonal damage, which may not be reflected by subjective explorations. Thus, 60% of patients with normal visual fields in our study had abnormal RNFL thickness measurements by OCT at the six-month visit [6]. Pueyo et al. enrolled 40 patients with multiple sclerosis who had normal VA and visual fields in a prospective cohort. Although the former examinations were normal, significant differences with healthy subjects were observed in Ishihara color tests and in most RNFL measurements provided by OCT. Comparisons with the normative database showed RNFL defects in 12 eyes (30%) [17].

Low contrast letter acuity (LCLA) is being increasingly used now as a visual outcome measure in MS and ON studies. Talman et al. demonstrated that progressive RNFL thinning occurs as a function of time in MS and is associated with clinically significant visual loss by low-contrast letter acuity. They found that visual loss by the 2.5% contrast chart was significantly associated with RNFL thinning. Scores from the 1.25% contrast chart, however, correlated less well with RNFL loss [18]. Fisher et al. found that lower visual function scores were associated with reduced average overall RNFL thickness. For every 1-line change in low-contrast letter acuity and in contrast sensitivity scores, RNFL thickness differences of 4 *μ*m on average were noted, accounting for age. Spearman rank correlations between overall average RNFL thickness and visual function scores were highly significant yet modest in magnitude, suggesting that visual dysfunction may occur in some patients in the absence of (or perhaps in advance of) RNFL axonal loss (Spearman *r* [*r*s] = 0.33 and *P* < .0001 for low-contrast letter acuity, *r*s = 0.31 and *P* < .0001 for contrast sensitivity, *r*s = 0.26 and *P* = .0005 for high-contrast VA) [10]. 

Thus, both LCLA and RNFL thinnings are being introduced as surrogate markers for disability in MS trials. However, it should be taken into account that some patients may present with visual loss even in the presence of a preserved RNFL thickness, while on the other hand patients with decreased RNFL thickness may not present severe dysfunction if nerve fiber loss does not affect the papillo-macular bundle. Furthermore, patients with visual loss adapt with time to their scotomas, so that visual function may improve as they learn to manage with their limitations. 

## 3. Optical Coherence Tomography in Patients with Clinically Isolated Syndrome

The development of a clinically isolated syndrome (CIS) represents the earliest clinical stage of multiple sclerosis. Outteryck et al. studied 56 patients with CIS, 18 with optic neuritis, and 38 without it. Two-thirds of the patients had dissemination in space according to the Barkhof criteria. All of the patients had a normal overall RNFL thickness. However, 14 patients (25%) and 7 controls (22%) had RNFL atrophy in at least 1 quadrant, according to the OCT database (Figure 3). There was no link between atrophy in 1 or more quadrants of the RNFL and dissemination in space according to the Barkhof criteria at initial MRI, nor with multifocal presentation, alteration of visual evoked potentials, or development of multiple sclerosis after 6 months according to the revised McDonald criteria [19]. However, the relationship between RNFL thinning in CIS and progression to MS is still unclear, since only long-term followup will determine if these changes are clinically relevant. 

## 4. Multiple Sclerosis

In the absence of optic neuritis, retrograde trans-synaptic retinal ganglion cell degeneration due to multiple sclerosis lesions within the posterior optic pathways could cause RNFL loss. Progressive axonal loss could also explain the RNFL thinning found in eyes of patients with multiple sclerosis without a history of optic neuritis (Table 2) [14]. In these eyes, mean RNFL loss is milder (7.08 *μ*m) than in eyes that have suffered optic neuritis (20.38 *μ*m) [2]. Some studies have only found a significant difference in eyes with and without optic neuritis for the temporal quadrant [20].

On average, 10 *μ*m differences in RNFL thickness are associated with 0.20 mm^3^ reductions in total macular volume. Eyes of patients with multiple sclerosis both with and without optic neuritis showed similar degrees of total macular volume reduction [21]. 

A moderate correlation has been found between RNFL thickness and the time from diagnosis of multiple sclerosis [11, 14, 22, 23]. However, the correlation with neurological disability quantified by the Expanded Disability Status Scale (EDSS) is less consistent: some authors have found a significant correlation between the EDSS and RNFL thickness [15, 22, 24, 25], while others have not [17, 26]. The strongest correlation was found in relapsing remitting MS (RRMS) [23]. The differences between these studies may be due to differences in the neurological status among study populations. It has been proposed that OCT may be more optimally used in little or moderately affected patients [13, 23]. 

RNFL thinning is greater when multiple sclerosis patients suffer an optic neuritis [21, 24], and more pronounced in the temporal quadrant (Table 2) [27]. No differences were detected between unaffected eyes of patients with multiple sclerosis with or without an eye affected of optic neuritis [22, 27]. When the RNFL is measured in patients who have suffered optic neuritis, the thinning is greater in patients with multiple sclerosis than when it constitutes a clinical isolated syndrome, and the difference is significant for the temporal quadrant [23]. This suggests that the disease process underlying multiple sclerosis increases the damage produced by an inflammatory episode. 

### 4.1. Macular Edema

Optical coherence tomography has become the most useful tool for the diagnosis of macular edema. This is not a common isolated manifestation; however, it could appear in multiple sclerosis patients with intermediate uveitis or as a side effect of therapies.

### 4.2. Recurrent Episodes of Optic Neuritis in Patients with Multiple Sclerosis

Costello et al. compared eyes with isolated optic neuritis to eyes with recurrent episodes of patients with different forms of MS and found an additional thinning when the inflammation recurs [23]. They conclude that the majority of patients may recover visual function after an isolated optic neuritis event because they do not suffer enough axonal damage to result in permanent visual impairment. Patients with severe or recurrent optic neuritis, however, may be at a greater risk of losing so many axons that they fall under the threshold required for complete visual recovery, thus increasing the likelihood that they will experience persistent visual defects [23]. 

### 4.3. Relationship with MRI Findings

Magnetic resonance image findings are currently considered the most sensitive and reliable markers for assessing inflammatory and axonal pathology in patients with multiple sclerosis. Conventional techniques are designed to be largely sensitive to inflammation (T2-weighted lesions) and not specifically reflect axonal damage with only modest correlation with clinical disability [25]. Alternatively diffuse brain atrophy has been linked with disability progression in multiple sclerosis [25]. Significant associations have been shown between the RNFL thickness and several MRI findings characteristic of brain atrophy:

- brain parenchymal fraction (which computes the volumes of various intracranial compartments and total brain parenchyma) [22, 25, 28],
- diffusion tensor imaging values [29],
- gray matter [22, 24] and white matter volume [24],
- increase in cerebrospinal fluid volume [25],
- magnetization transfer ratio [29],
- T1-lesion volumen [22].

Frohman et al. studied twelve patients with multiple sclerosis and found that low contrast visual acuity, RNFL thickness, and optic nerve radius were the variables with the highest predictive value in discerning differences between healthy controls and patients. Both the radius of the affected eyes and its fractional anisotropy predicted the RNFL of the affected eye; however, the RNFL thickness was the only independent predictor of lower contrast sensitivity. T1 and T2 lesion volumes, measures of optic nerve atrophy, and measures of grey matter atrophy were related to RNFL thickness, however, they explained only about 20% of variance [29]. 

In multiple sclerosis patients without optic neuritis, axonal loss seems to correlate better with MRI parameters than in those that have suffered optic neuritis [22]. RNFL thickness correlates with brain atrophy more strongly in RRMS than in secondary progressive multiple sclerosis (SPMS). This might be due to a basement effect in the progressive group, in which RNFL or brain tissue may have reached their lowest levels so that further damage is almost impossible. Another possibility is that most patients with SPMS have clinical decline due to cumulative spinal cord disease rather than accumulation of brain disease [25]. Macular volume does not correlate with MRI features [25].

### 4.4. Types of Multiple Sclerosis

There seem to be different patterns of axonal loss among the different types of multiple sclerosis according to their clinical course (Table 3). Henderson et al. studied patients with progressive forms of multiple sclerosis, excluding those who had suffered optic neuritis in both eyes. Axonal loss was significant compared to controls, for the mean RNFL in the SPMS group and for the temporal quadrant in both progressive forms (53.6 *μ*m, SD 13.2 *μ*m and 63.7 *μ*m, SD 14.6 *μ*m, for SPMS and primary progressive (PPMS] types, resp.). The only difference found between both groups was the thinner temporal quadrant in the SPMS group [40]. These results could be explained by subclinical optic neuritis attacks suffered by SPMS patients in the remittent recurrent phase, by differences in the time from diagnosis that existed between both groups or due to distinctive preferences in the nervous system affected in each form [40].

Pulicken et al. also found RNFL thinning in the progressive forms, which was more pronounced than in patients with RRMS [37], and Siepman et al. did not find significant differences when comparing eyes of patients with PPMS and RRMS [13]. Therefore, it seems that during the progressive phase progressive axonal loss also develops, being more pronounced in the SPMS type [37].

Costello et al. studied patients who had had isolated optic neuritis (without a diagnosis of MS) and patients who had had an episode of neuritis and were already diagnosed with RRMS, SPMS, or PPMS. Optic atrophy was more severe in the secondary progressive group with more pronounced differences in the temporal quadrant. The differences among multiple sclerosis types are more difficult to appreciate in eyes without optic neuritis [23].

Total macular volumes also differed between multiple sclerosis disease subtypes, with lower values seen in SPMS [mean (SD], 6.25(0.52] mm^3^) than in PPMS (mean (SD), 6.57(0.50] mm^3^) [21]. 

### 4.5. Visual Prognosis

Multiple sclerosis patients have worse contrast sensitivity and visual fields if they have suffered an episode of optic neuritis, in accordance with their decreased RNFL thickness, than if they just have subclinical axonal loss [10, 32, 41].

Visual prognosis after an episode of optic neuritis is good, since approximately three out of four patients retain a visual acuity of 20/20 after 15 years [42]. Visual acuity after an episode of neuritis is similar in patients already diagnosed with multiple sclerosis to patients in whom it is an isolated manifestation. However, visual field mean deviation, a parameter that measures light sensibility depression, is slightly lower for multiple sclerosis patients [32], probably because visual acuity is less sensitive to asses visual function in multiple sclerosis patients than other examinations, such as color vision, stereopsis, or contrast sensitivity [8, 43].

Visual acuity in patients with multiple sclerosis without optic neuritis does not differ from healthy controls. However, when tests that explore spatial (Sloan and Pelli-Robson charts) and temporal (frequency doubling technology perimetry) contrast sensitivity are employed, visual function is found to be worse in multiple sclerosis patients when compared to control subjects [31]. In their study, Merle et al. found that eyes with a previous history of optic neuritis presented an important decrease in RNFL thickness, which was correlated with the results of all the visual function tests performed, including VA [31].

Visual fields may be normal even if RNFL loss is detected: Cheng et al. found no perimetric defects in 4% patients with mean RNFL atrophy and in 18% with at least sectorial atrophy according to normative data [38]. Disagreement between RNFL thickness and visual fields is probably influenced by cognitive dysfunction or slowed reaction times during subjective field testing, which can interfere with decision-making, in patients with multiple sclerosis and also by central visual pathway damage that does not result in retrograde degeneration. However, when functional loss is worse than −10 dB, the authors concluded that it is better to use mean deviation for monitoring disease progression, because RNFL loss has almost reached a plateau at approximately 60 *μ*m (Figure 4) [38].

Lower RNFL values have been correlated with reduced visual acuity and mean deviation. Every 10 *μ*m decrease in RNFL correlated with a 5.8 dB decrease in visual field sensitivity and a 0.46 reduction in visual acuity for RNFL values below 75 *μ*m [23]. 

### 4.6. Evolution

Longitudinal studies have been performed to assess changes in RNFL thickness. Talman et al. followed 299 patients with multiple sclerosis for at least six months, with a median followup of 18 months, ranging between 6 months and four and a half years. They found that each year of followup was associated on average with a 2.0 *μ*m decreases in RFNL thickness. This rate of axonal loss was similar in patients with and without a history of optic neuritis. Eyes with visual loss by low-contrast letter acuity and VA (measured with an ETDRS chart and concerted to logMAR for analysis) had greater degrees of RNFL thinning during followup compared to those without visual changes. RNFL thinning was also associated with progressive changes in neurological impairment measured by the EDSS [18]. Sepulcre et al. found a decrease in average RNFL thickness of 4.8 *μ*m in patients after 2 years. They found that patients with more active disease have a thinner temporal quadrant RNFL compared with stable patients. Patients with new relapses during followup had a thinner RNFL in the temporal quadrant than relapse-free patients by the end of the study [24]. García-Martín et al. enrolled 81 patients with a diagnosis of defined multiple sclerosis: 31 of the patients (38.3%) received no specific treatment, whereas the other 50 patients (61.7%) were treated with interferon beta. Most studied eyes (75.3%) were from patients without a history of optic neuritis. Statistically significant differences were observed between the baseline and 1-year examinations in all the RNFL thickness measurements and macular volume and in VA (logMAR), whereas perimetry results revealed no differences between treated and untreated patients. The greatest decrease was found in the average and the inferior OCT RNFL thickness (of 3%), with a baseline mean of 90.46 *μ*m and 115.46 *μ*m versus 85.96 *μ*m and 109.12 *μ*m at the 1-year followup, respectively, No correlation was found between the 1-year change in EDSS and RNFL measurements. They concluded that axonal loss in the optic nerve of patients with multiple sclerosis is far greater than that which occurs in healthy subjects, regardless of the presence of a history of optic neuritis [44].

## 5. Neuromyelitis Optica

Visual prognosis is much worse if optic neuritis occurs in patients with neuromyelitis optica. Only one episode is capable of producing legal blindness in almost one third of patients and only about 45% of them completely recover visual function [47]. An ischemic vascular mechanism has been proposed in its pathogenesis to explain at least partially its severity [48]. Ratchford et al. have suggested that an RNFL thickness loss after an episode of optic neuritis of more than 15 *μ*m may be considered a marker for this disease instead of multiple sclerosis, together with the absence of a visual improvement of at least two lines [49]. Naismith et al. estimated that for every 1 *μ*m decrease in the RNFL thickness, the odds of being diagnosed with NMO increased by 8% [26]. Several reports have confirmed that axonal loss after an episode of optic neuritis in patients with neuromyelitis optica is greater than in patients with multiple sclerosis (Table 4) [45, 46]. This difference persisted even after adjusting the RNFL for visual outcome [26]. It has also been shown that the superior and inferior quadrants are more intensely affected after NMO, so that the pattern of the RNFL loses its characteristic humps [26, 45]. Recurrent episodes of optic neuritis lead to further RNFL loss [45].

The mean RNFL thickness of the unaffected fellow eye in NMO has been found to be greater than the unaffected multiple sclerosis eyes. This sparing of the unaffected felloe eye in NMO compared to MS may be explained by a more common occurrence of subclinical optic neuritis in multiple sclerosis: axonal attrition in multiple sclerosis independent of optic neuritis or an increased predilection of multiple sclerosis lesions in the optic chiasm or tracts [26].

As in multiple sclerosis, mean RNFL is correlated with best-corrected visual acuity. Studies agree on the fact that there is a critical value of RNFL thickness below which further decreases of the RNFL lead to incomplete visual recovery. This critical value has been set at 71.41 *μ*m [45]. Below 50–52 *μ*m, vision drops to ≤20/100 [26, 46]. 

In a retrospective study, Nakamura et al. evaluated the effects of high dose intravenous methyl-prednisolone on the outcomes after optic neuritis in patients with neuromyelitis optica. Early treatment, especially within 3 days after onset, led to a greater probability of preserving an RNFL > 71.41 *μ*m (the cutoff point in this study for preserving a visual acuity >20/20) [45]. 

Even if RNFL loss is greater in NMO as compared to MS, at each level of visual function there was a considerable overlap in OCT measures, limiting the role of OCT to differentiate the two conditions on an individual basis (Figure 5) [50]. 

## 6. Conclusions

- Optical coherence tomography confirms the presence of optic disc edema in anterior neuritis, reflected as a thickening of the RNFL.
- Axonal atrophy develops after optic neuritis so that six months after the event, the RNFL thickness is predictive of visual and neurological disability. However, it may be more optimally used in little or moderately disable patients.
- Optical coherence tomography can detect subclinical axonal loss in patients with normal visual acuity and visual fields. Contrast sensitivity seems to be the most useful test to detect subtle visual impairment.
- The temporal quadrant is the most vulnerable to the disease process.
  - Temporal RNFL thickness may be decreased as soon as two months after the event.
  - Reduced temporal thickness is often the only sign that may differentiate multiple sclerosis patients from healthy subjects and between primary and secondary progressive forms.
  - It may provide important insights regarding relapse related activity in multiple sclerosis patients.
- During the progressive phases of multiple sclerosis, axonal loss also occurs at the optic nerve; this axonal loss is detected by OCT as RNFL loss and is greater in the SPMS type.
- When multiple sclerosis patients are followedup, an approximate decrease of 2 *μ*m in RFNL thickness is detected per year. Progressive changes seem to correlate with changes in neurological impairment measured by the EDSS.
- Brain atrophy is at least moderately correlated to RNFL thickness and multiple sclerosis patients have decreased RNFL thickness even without a history of optic neuritis. These results suggest that the RNFL thinning reflects pathology that extends beyond local injury to the optic nerve by optic neuritis.
- A stronger correlation with MRI results is unlikely since axons are not the only component of the brain and because brain atrophy also reflects synaptic changes, loss of myelin, gliosis, and changes in water content.
- Visual prognosis is much worse if optic neuritis occurs in patients with neuromyelitis optica, which leads to a more sever thinning of the RNFL when compared to optic neuritis in multiple sclerosis patients.
- OCT thus seems to be a promising outcome measure for neuroprotective trials. However, overall RNFL thickness is not always directly correlated with visual function and measuring both mean RNFL thickness and temporal RNFL thickness (usually more related to visual acuity) would require more patients to be included into the studies. Furthermore, it may be difficult to distinguish axonal loss related to age with axonal loss due to the disease process in MS. The relationship between axonal loss and OCT is not clear: future studies need to evaluate it.

## Figures and Tables

**Figure 1:** Fundus photograph, visual fields, and optical coherence tomography of a 30-year-old man who consulted due to ocular pain and visual loss in his left eye for two weeks. Optical coherence tomography shows an increased retinal nerve fiber layer thickness in his left eye due to optic nerve edema.

**Figure 2:** Patient who developed retrobulbar neuritis in his right eye as an initial clinically isolated syndrome. In only three months, axonal loss can be detected in the eye that suffered the neuritis.

**Figure 3:** Patient who suffered a motor clinical isolated syndrome and fulfilled Barkhof's magnetic resonance imaging criteria. Optical coherence tomography shows a decreased retinal nerve fiber layer in both eyes (more intense in the right eye) even without a history of optic neuritis.

**Figure 4:** Patient with multiple sclerosis and severe bilateral RNFL thinning with history of optic neuritis. SD-optical coherence tomography analysis found no further loss during a year.

**Figure 5:** Teenager diagnosed of neuromyelitis optica who has suffered bilateral optic neuritis as well as myelitis. Although normative data are not available, the retinal nerve fiber layer thickness measured with optical coherence tomography is extremely low.

**Table 1:** Comparison of RNFL thickness (*μ*m) between both eyes of patients who have suffered unilateral optic neuritis and healthy control subjects. Values are expressed as mean (standard deviation).

	Patients	ON eye	Fellow eye	Control
Outteryck et al.[19]	Non-MS	92.27 (12.82)	—	98.71 (9.08)
Grazioli et al. [28]	MS	81.7 (19.2)	93.6 (15.3)	—
Klistorner et al. [9]	MS and non-MS	84.5 (15. 1)	103.8 (10.8)	104.0 (9.2)
Siger et al. [22]	MS	83.92 (17.63)	91.08 (19.3)	—
Costello et al. [7]	Non-MS	86.1	101.6	—
Noval et al. (data not published)	MS and non-MS	84.95 (23.45)	103.40 (15.27)	105.5 (10.51)
Fisher et al. [10]	MS	85 (17)	96 (14)	105 (12)
Costello et al. [5]	Non-MS	77.5 (29.87)	99.8 (32.5)	—
Trip et al. [11]	MS and non-MS	68.7 (18.8)	94.6 (14.9)	102.9 (14.6)
Parisi et al. [12]	MS	59.79 (10.80)	82.73 (10.73)	111.11 (11.42)

MS: multiple sclerosis.

NON: MS healthy subjects.

ON: optic neuritis.

**Table 2:** Comparison of RNFL thickness (*μ*m) between both eyes of patients diagnosed of multiple sclerosis who have suffered unilateral optic neuritis and healthy control subjects.

	MS with ON	MS without ON	Control
Siepman et al. [13]	72.2 (14.4)	89.5 (14.2)	—
Khanifar et al.* [14]	83.0 (14.0)	90.5 (13.2)	97
Costello et al. [23]	79.5 (18.8)	97.0 (14.3)	—
Bock et al. [27]	86.2 (16.2)	97.0 (13.1)	105.2 (9.4)
Quelly et al. [30]	78.01 (17.43)	95.24 (11.64)	—
Merle et al. [31]	80.81 (18.4)	96.7 (15.8)	106 (12.2)
Oreja-Guevara et al. [32]	76.42 (16.87)	89.45 (17.68)	—
Frohman et al. [33]	70.3 (13.4)	101.8 (6)	101.9 (8.9)
Burkholder et al. [21]	85.7 (19.0)	95.6 (14.5)	104.5 (10.7)
Spain et al. [34]	75.81	90.93	—
Siger et al. [22]	83.92 (17.63)	94.38 (15.0)	100.3 (12.1)
Pueyo et al. [35]	84.46	94.20	104.97
Zaveri et al. [36]	81.8 (19.3)	95.6 (15.0)	104.6 (10.3)
Pulicken et al. [37]	84.2 (14.7)	95.9 (14)	102.7 (11.5)
Gundogan et al. [20]	—	107.6 (16.3)	110.9 (10.3)
Cheng et al. [38]	76.12 (14.92)	96.45 (11.73)	—
Fisher et al. [10]	85 (17)	96 (14)	105 (12)

*Heidelberg Spectralis. Value for normals taken from normative database.

MS: multiple sclerosis.

ON: optic neuritis.

**Table 3:** Comparison of RNFL thickness (*μ*m) among different types of multiple sclerosis.

		RRMS	SPMS	PPMS	Control
Albrecht et al. [39]		86.91 (21.51)	70.57 (16.76)	80.45 (17.76)	103.4 (10.96)
Henderson et al. [40]	Non-ON	Not supplied	88.4 (10.9)	Not supplied	Not supplied
Pulicken et al. [37]		94.4 (14.6)	81.8 (15.6)	88.9 (13.3)	—

RRMS: recurrent remittent multiple sclerosis.

SPMS: secondary progressive multiple sclerosis.

PPMS: primary progressive multiple sclerosis.

**Table 4:** Comparison of RNFL thickness (*μ*m) between multiple sclerosis and neuromyelitis optica.

	NMO ON eye	NMO fellow eye	MS ON eye	MS fellow eye	Control
Nakamura et al. [45]	63.84 (23.47)	106.36 (14.55)	84.28 (14.18)	109.45 (12.78)	—
Naismith et al. [26]	54.8 (3.7)	—	76.5 (2.4)	—	—
Merle et al. [46]	65.44 (24.19)		83.85 (24.12)		106.24 (12.46)

MS: multiple sclerosis.

NMO: neuromyelitis optica.
